# Synovitis Ointment Improved Knee Osteoarthritis by Suppressing SDF-1/CXCR4 Signaling Pathway

**DOI:** 10.1155/2022/7719301

**Published:** 2022-07-01

**Authors:** Jin Zhang, Min Zhao, Jing Liu, Ke Wang, Xiang Cai, Wei Xiao, Le Wang, Mang Wang, Lei Zhang, Chi Zhang

**Affiliations:** ^1^Department of Orthopedic, Wuhan Hospital of Traditional Chinese Medicine, Wuhan 430014, China; ^2^Department of Acupuncture, Wuhan Hospital of Traditional Chinese Medicine, Wuhan 430014, China; ^3^Department of Surgery, Wuhan Hospital of Traditional Chinese Medicine, Wuhan 430014, China

## Abstract

**Objective:**

Knee osteoarthritis (KOA) remains a challenge for clinicians worldwide and lacks major advancements in treatment. In this study, we investigated the mechanism of synovitis ointment interference on KOA.

**Methods:**

SD rats were used to establish KOA models and were randomly divided into five groups: the control group, the KOA group, the KOA + synovitis ointment group, the KOA + Western medicine group, and the KOA + Chinese medicine group. Detection of pathological injury of the joint was observed through HE staining. Enzyme-linked immunosorbent assay (ELISA) was used to measure the expression of SDF-1, CXCR4, MMP-9, and MMP-13. Effects of synovitis ointment on bone cell fibrosis were detected through Masson staining, and the relative mRNA expression of PLOD2, COL1A1, TIMP1, and TGF-*β* was observed using the real-time quantitative (RT-PCR) method.

**Results:**

Mankin's score and the knee diameters showed that the KOA model has been successfully established; compared with the OA group, the synovitis ointment group improved the pathological injury of the knee joint. Compared with the KOA group, the synovitis ointment group, the KOA + Western medicine group, and the KOA + Chinese medicine group significantly decreased the expression of SDF-1, CXCR4, MMP-9, and MMP-13. Synovitis ointment reduced the relative content of bone cell fiber compared to that in the KOA group. While, the relative mRNA expression of PLOD2, COL1A1, TIMP1, and TGF-*β* was significantly decreased in the synovitis ointment group.

**Conclusion:**

Synovitis ointment inhibited the inflammation and bone cell fibrosis of KOA, and the mechanism was related to the SDF-1/CXCR4 singling pathway.

## 1. Introduction

Knee osteoarthritis (KOA) is one of the joint degenerative diseases leading to disability in the elderly [1]. Its incidence is increasing year by year and the patient have the tendency of being younger, which seriously threatens the health of humans and the quality of life [2, 3]. As the pathogenesis and etiology of KOA are still inaccurate, it is difficult to obtain satisfactory results in the clinical treatment of KOA. Previous studies have shown that cartilage damage could cause synovial inflammation, and chondrocyte-mediated inflammation played a key role in the occurrence and development of osteoarthritis [4]. Therefore, effective inhibition of inflammation might have a great significance in delaying or even reversing the process of the KOA.

Chemokine SDF-1 (CXCL12) is a cytokinin bound to a specific G protein-coupled receptor (CXCR4; CD184) and plays an important role in physiological and pathological processes [5, 6]. Studies have shown that in patients with KOA, the SDF-1/CXCR4 pathway was involved in maintaining or promoting the inflammatory process [7]. It affected the proliferation of blood vessels through MMPs, promoted cell proliferation and migration, inhibited cell apoptosis, and promoted inflammation-driven colorectal cancer [8, 9]. Meanwhile, bone cell fibrosis was an important indicator in the development of KOA [10]. PLOD2, COL1A1, TIMP1, and TGF-*β* were generally considered fibrosis markers [11]. Thus, inhibiting inflammation and bone cell fibrosis may be a potential method for the treatment of KOA.

In recent years, traditional Chinese medicine had a significant effect on KOA, which could effectively reduce the risk of total knee replacement [12]. Studies had shown that Fang Sheng Yu decoction combined with Wu Ling powder [13] and Tian Nan Xing decoction combined with Bu Shen Huo Xue decoction could relieve the pain in knee joint and improve the function of the knee joint [14, 15]. Synovitis ointment was made with Radix Aconiti Konii, Radix Aconiti, Radix Noctis, Kaschin, Kaempferi, Hyacinth, *Asarum*, and Baijiu. It had the functions of anti-inflammatory and analgesic, expelling wind and cold, promoting blood circulation, and removing dampness. The direct external application could reduce inflammation and analgesia and repair the synovium of cartilage tissue. In the long-term clinical treatment of KOA, synovitis ointment significantly ameliorated the symptoms of KOA and improved the health and quality of life. However, the specific mechanism of synovitis ointment on KOA is still unclear. In this study, through the animal experiment, the mechanism of KOA treated with synovitis ointment was studied, which provided a scientific basis for clinical application and improved the quality of life of the elderly. This was of great significance to improve the physical quality of the people and social development.

## 2. Materials and Methods

### 2.1. Experimental Animals

Thirty specific pathogen-free (SPF) male SD rats (200 ± 10 g, 6 weeks) were purchased from the China Three Gorges University (Hubei, China). Rats were fed at (22–26)°C with 12 h day/night cycle and free access to water and food for 7 d. All animal experiments confirmed to the relevant regulations of the Hubei Provincial Animal Management Committee's “Ethics Certificate for Experimental Animals.” The animal study protocol was approved (approval no: SYXK (E) 2018–0104). Experiments were conducted in accordance with the ethical guidelines of the Hubei Provincial Animal Management Commission (permit no. 42010200004453).

### 2.2. Establishment of the KOA Model

All rats were anesthetized by intraperitoneal injection of pentobarbital sodium at 40 mg/kg. A longitudinal incision (2 cm) was made on one side of the knee to expose the knee joint. Then, the meniscus on one side of the knee was removed, and a cotton ball was used to stop the bleeding. The incision was sutured with 5–0 silk thread. Finally, all the rats were normally fed and conducted treatment in the 6th week of modeling.

### 2.3. Animal Grouping

Rats were randomly divided into five groups: the control group, the KOA group, the KOA + synovitis ointment group, the KOA + western medicine group, and the KOA + Chinese medicine group. The KOA model was established for all rats except for the control group rats. In the KOA + synovitis ointment group, rats were treated with 5 g synovitis ointment for 6 hours per day on the knee joint. In the KOA + Western medicine group, rats were treated with 0.4 g diclofenac cream (Sino US Tianjin Shike Pharmaceutical Co., Ltd., Tianjin, China) for each of the knee joint every day for 6 hours. In the KOA + Chinese medicine group, rats were treated with 5 g Golden Powder Cream for 6 hours per day on the knee joint. All the KOA rats were treated for 4 weeks.

### 2.4. Synovitis Ointment and Golden Powder Cream

Synovitis ointment is made from 50 g of Aconiti Kusnezoffii Radix, 50 g of Aconiti Radix, 50 g of Arisaematis Rhizoma, 50 g of Nardostachyos Radix et Rhizoma, 50 g of Rhizoma Kaempferiae, 50 g of Corydalis Rhizoma, and 20 g of Asari Radix et Rhizoma. Collect the powder and add 3 times the mass of alcohol to stir into a plaster, and 5 g plaster was placed in gauze for treatment. Golden Powder Cream: in accordance with the records of Chinese Pharmacopoeia, Radix Trichosanthis (320 g), Angelicae Dahuricae Radix (160 g), Curcumae Longae Rhizoma (160 g), Rhei Radix et Rhizoma (160 g), Phellodendri Chinensis Cortex (160 g), Atractylodis Rhizoma (64 g), Magnoliae Officinalis Cortex (64 g), *Citrus reticulata* Blanco (64 g), Radix Rhizoma Glycyrrhizae (64 g), and Arisaematis Rhizoma (64 g) were ground into a fine powder and prepared into a paste with honey. The ratio of Golden Powder Cream and honey is 3:1.5 g plaster was placed in gauze for treatment.

### 2.5. Sampling and Tissue Preparation

Blood samples were collected from the abdominal aorta. Serum samples were obtained by centrifugation at 4°C. The bone tissues were cut into tissue blocks and then fixed with decalcification solution for 2 d. Next, the tissues were permeabilized by xylene, embedded with paraffin, and cut into 3 *μ*m sections, which were normally conducted in a 42°C water bath and dried.

### 2.6. HE Staining

The paraffin sections were dewaxed by xylene (Sinopharm Chemical Reagent Co., Ltd., Shanghai, China) and a series of ethanol (Sinopharm Chemical Reagent Co., Ltd., Shanghai, China). Then, HE staining was performed and observed under a microscope (Leica, Wetzlar, Germany).

### 2.7. Masson Staining

The paraffin sections were dehydrated and stained with a drop of hematoxylin staining solution and ferric chloride aqueous solution for 5 min and then differentiated with a drop of ethanol hydrochloride. The morphological changes in cartilage tissues were observed under a microscope.

### 2.8. Real-Time Quantitative (RT-PCR) Methods

100 mg tissue samples were put into TRIzol (Ambion, Shanghai, China) for mRNA extraction. The cDNA was obtained through a reverse transcriptase kit (TAKARA, Dalian, China) with gDNA remover. The relative mRNA expression of PLOD2-F, COL1A1, TIMP1, and TGF-*β* was performed in duplicate to determine an endogenous control of glyceraldehyde-3-phosphate dehydrogenase (GAPDH). The primer (Wuhan Tianyi Huayu Gene Technology Co., Ltd., Wuhan, China) sequences are given in Table 1.

### 2.9. Enzyme-Linked Immunosorbent Assay (ELISA)

The serum samples were collected and concentrations of MMP-9, MMP-13, SDF-1, and CXCR4 were measured by using specific rat enzyme-linked immunosorbent assay (ELISA) kits (Wuhan Beinlai Biotechnology Co., Ltd., Wuhan, China) as per the manufacturer's instructions.

### 2.10. Statistics

All data were expressed as mean ± SD and conducted using the SPSS 21.0 software. One-way analysis of variance (ANOVA) was used for comparisons between groups and *P* < 0.05 was considered statistically significant. Multiple comparisons between groups were performed using Student's *t*-tests. Histological analyses were performed by two experienced investigators who were double-blinded.

## 3. Results

### 3.1. Effects of Synovitis Ointment on Mankin's Score and Keen Diameter in the KOA Model

To investigate the effect of synovitis ointment on KOA development and progression, we observed the cartilage tissue damage of the knee joint through HE staining and measured the diameter of the knee joint in rats. In the control group (Figure 1(a)), no histological changes were observed. In contrast, severe damage in HE sections from the KOA group was observed (Figure 1(b)). Full-thickness cartilage defect and microfracture in the fibrocartilage were seen in this group. The KOA + synovitis ointment group (Figure 1(c)) showed lower levels of damage than that of the KOA group. Regarding Mankin's score and knee diameter (Figures 1(f)–1(g)), Mankin's score in control, KOA + synovitis ointment, KOA + Western medicine, and KOA + Chinese medicine groups were low, but high scores were observed in the KOA group. In addition, the knee diameters in the KOA group were significantly higher than that of other groups (*P* < 0.05). This demonstrated that synovitis ointment was favorable to KOA recovery.

### 3.2. Effects of Synovitis Ointment on the Expression of SDF-1, CXCR4, MMP-9, and MMP-13

To unravel the effects of synovitis ointment on SDF-1/CXCR4, we examined the expression of SDF-1, CXCR4, MMP-9, and MMP-13 in serum under different treatment conditions through the ELISA method (Figure 2). The levels of SDF-1, CXCR4, MMP-9, and MMP-13 were higher in the KOA group than those in groups with drug treatment. This finding confirmed that synovitis ointment was likely to suppress the osteoarthritis of the knee inflammation through downregulating the SDF-1/CXCR4 signaling pathway.

### 3.3. Effects of Synovitis Ointment on Bone Cells Fibrosis

To determine the effect of synovitis ointment on bone cells fibrosis, Masson staining was used for the cartilage collagen fiber staining. In the KOA group (Figure 3(b)), brighter and wider area blue was observed when compared to the control group (Figure 3(a)). The application of synovitis ointment caused significant reduction in the formation of bone cell fibrosis (Figure 3(c)). These results indicated that synovitis ointment was able to inhibit the increase of bone cell fibrosis.

### 3.4. Effects of Synovitis Ointment on the Relative mRNA Expression of PLOD2, COL1A1, TIMP1, and TGF-*β*

To verify the effects of synovitis ointment on bone cells fibrosis, through RT-PCR assays, we examined the relative mRNA expression of PLOD2, COL1A1, TIMP1, and TGF-*β* under different treatment conditions (Figure 4). The levels of PLOD2, COL1A1, TIMP1, and TGF-*β* were significantly higher in those lacking drug treatments than those treated with synovitis ointment (*P* < 0.05). This further proved that synovitis ointment treated osteoarthritis of the knee through inhibiting osteocytes fibrosis.

## 4. Discussion

KOA is known as a chronic degenerative disease and a significant public health problem, which has become one of the main reasons affecting the elderly life quality [16]. At present, there are several methods for treatment of KOA such as nonspecific anti-inflammatory, electrotherapy, acupuncture, Chinese medicine, intraarticular injection of drugs, and weight loss and psychotherapy. Among them, traditional Chinese medicine synovitis ointment in the treatment of KOA has its unique curative effect. But its specific mechanism of action is rarely involved and not specific in-depth. In this study, we removed the meniscus of the knee to construct the model of KOA and confirmed it was constructed successfully through Mankin's score. Rats knee transverse diameter and HE results showed synovitis cream could effectively alleviate the symptoms of KOA.

SDF-1 is a member of CXCL12 chemokine family, which is secreted by many kinds of cells and has chemotactic and proliferative effects. It is regarded as a specific index of inflammatory response. CXCR4, as its specific receptor, is a G protein-coupled receptor, which is mainly expressed in immune cells and plays an important role in cell growth and development [17]. As a pair of important inflammatory response chemokines, the SDF-1/CXCR4 signaling pathway plays an important role in the occurrence and development of KOA [18]. MMP-9 and MMP-13 are important members of the matrix metalloproteinase (MMP) family. MMP-13, known as collagenase-13, plays a regulatory and pivotal role in the cascade of activation of MMPs. It is not only regulated by a variety of MMPs factors but also participates in the degradation process of ECM after activation. MMP-9 is a gelatinase, and activated MMP-9 can directly degrade ECM and promote the occurrence and development of physiological and pathological osteolysis. It was widely believed that MMPs are involved in the occurrence and development of cartilage degenerative changes, and MMP-13 and MMP-9 play an important role in the degradation of cartilage extracellular matrix [19]. In this study, we found that the expression levels of SDF-1, CXCR4, MMP-9, and MMP-13 in KOA rats increased, which is consistent with reports in the literature. After applying with synovitis ointment, the expression levels of SDF-1, CXCR4, MMP-9, and MMP-13 reduced significantly in KOA rats. These results indicated that the mechanism of synovitis ointment alleviating knee arthritis is related to reducing the expression of SDF-1, CXCR4, MMP-9, and MMP-13.

KOA is most likely to invade articular cartilage during its occurrence and development. Cartilage damage and degeneration are one of the important signs of KOA. Before early morphologic changes in articular cartilage, different degrees of synovitis can be observed including synovial edema, hyperplasia, and fibrosis [20]. Synovial inflammation and articular cartilage damage interact and influence each other during KOA. Articular cartilage wear particles, and other degradation products can induce macrophage-like synovial cells to swallow and remove these debris, stimulate the inflammation of the surrounding synovial tissue, promote the secretion of joint fluid from fibroblast-like synovial cells, and cause joint swelling [21]. Hence, we measured the levels of fibrosis markers PLOD2, COL1A1, TIMP1, and TGF-*β* in bone tissue through RT-PCR. In the KOA groups, PLOD2, COL1A1, TIMP1, and TGF-*β* levels were increased. As expected, synovitis ointment decreased the levels of PLOD2, COL1A1, TIMP1, and TGF-*β*. Studies suggested that synovitis ointment could reduce arthritis inflammation through reducing synovial fibrosis.

## 5. Conclusion

Synovitis ointment reduces the expression of SDF-1, CXCR4, MMP-9, and MMP-13 in rats with KOA, decreases the increase of knee joint diameter, alleviates KOA injury, inhibits the expression of PLOD2, COL1A1, TIMP1, and TGF-*β* mRNA to prevent osteoblast fibrosis, and finally promotes knee joint recovery. The target of synovitis cream is related to osteoclast fibrosis. In the future, we will conduct further research on the inhibition of osteoclast fibrosis by synovitis ointment and expect to discover and prove the target of synovitis ointment for the treatment of KOA.

## Figures and Tables

**Figure 1:** Mankin's score and knee diameter of joint tissue in the KOA model. The HE staining of joint tissue. (a) The control group. (b) The KOA group. (c) The KOA + synovitis ointment group. (d) The KOA + Western medicine group. (e) The KOA + Chinese medicine group. Mankin's score (f) and knee diameter (g) of joint tissue.

**Figure 2:** The expression of MMP-9 (a), MMP-13 (b), SDF-1 (c), and (d) CXCR4 in serum. The results are presented as the mean ± SD, *n* = 6. ^∗^P<0.05 vs. control.

**Figure 3:** The Masson staining of joint tissue in the KOA model. (a) The control group. (b) The KOA group. (c) The KOA + synovitis ointment group. (d) The KOA + Western medicine group. (e) The KOA + Chinese medicine group.

**Figure 4:** The relative mRNA expression of PLOD2 (a), COL1A1 (b), TIMP1 (c), and TGF-*β* (d) of joint tissue in KOA rats. The results are presented as the mean ± SD, *n* = 6. ^∗^P<0.05 vs. control.

**Table 1:** The primer sequences.

Gene	Primer sequences	Product length (bp)
PLOD2-F	GAACATTACGGCAAGTGGT	192
PLOD2-R	GGCAAATCCCTTGGTGTA	
COL1A1-F	AGATGTCCTATGGCTATGATGAG	288
COL1A1-R	CTGTTCCAGGCAATCCAC	
TIMP1-F	GGCATCCTCTTGTTGCTATCATT	281
TIMP1-R	CTGCGGTTCTGGGACTTGTG	
TGF-*β*-F	ACCGCAACAACGCAATCTAT	206
TGF-*β*-R	ACCAAGGTAACGCCAGGAAT	
GAPDH-F	CAAGTTCAACGGCACAG	138
GAPDH-R	CCAGTAGACTCCACGACAT	

## Data Availability

The data used to support the findings of this study are available from the corresponding author upon request.
